The article "Expression of adrenomedullin in human colorectal tumors and its role in cell growth and invasion in vitro and in xenograft growth in vivo" was retracted in 2024. Reasons: duplicated images; unreliable data; unreliable results or conclusions.

# Expression of adrenomedullin in human colorectal tumors and its role in cell growth and invasion in vitro and in xenograft growth in vivo

**DOI:** 10.1002/cam4.51

**Published:** 2013-01-29

**Authors:** Emilie Nouguerède, Caroline Berenguer, Stéphane Garcia, Bahia Bennani, Christine Delfino, Isabelle Nanni, Laetitia Dahan, Mohamed Gasmi, Jean-François Seitz, Pierre-Marie Martin, L'Houcine Ouafik

**Affiliations:** 1 Inserm, UMR 911-CRO2Marseille, F-13000, France; 2 Laboratoire d'Anapathologie, CHU Nord (AP-HM)Marseille, F-13000, France; 3 Laboratoire de Biologie du Cancer, Faculté de Médecine et de PharmacieBP 1893, Route de Sidi Harazem, Fès, Maroc; 4 Laboratoire de Transfert d'Oncologie Biologique (AP-HM)Marseille, F-13000, France; 5 Service d'oncologie digestive, CHU la Timone (AP-HM)Marseille, F-13000, France; 6 Service de Gastro-entérologie, CHU Nord (AP-HM)Marseille, F-13000, France

**Keywords:** Adrenomedullin, AM_1_ and AM_2_ receptors, angiogenesis, colorectal cancer, tumor growth

## Abstract

Adrenomedullin (AM) is a multifunctional peptide vasodilator that transduces its effects through calcitonin receptor-like receptor/receptor activity-modifying protein-2 and -3 (CLR/RAMP2 and CLR/RAMP3). In this study, real-time quantitative reverse transcription demonstrated a significant expression of AM mRNA in tumor samples from colorectal cancer (CRC) patients in clinical stage II, III, and IV when compared with normal colorectal tissue. AM, CLR, RAMP2, and RAMP3 proteins were immunohistochemically localized in the carcinomatous epithelial compartment of CRC tissue. Tissue microarray analysis revealed a clear increase of AM, CLR, RAMP2, and RAMP3 staining in lymph node and distant metastasis when compared with primary tumors. The human colon carcinoma cells HT-29 expressed and secreted AM into the culture medium with a significant increase under hypoxia. Treatment of HT-29 cells with synthetic AM stimulated cell proliferation and invasion in vitro. Incubation with anti-AM antibody (αAM), anti-AM receptors antibodies (αAMR), or AM antagonist AM_22–52_ inhibited significantly basal levels of proliferation of HT-29 cells, suggesting that AM may function as an autocrine growth factor for CRC cells. Treatment with αAM significantly suppressed the growth of HT-29 tumor xenografts in vivo. Histological examination of αAM-treated tumors showed evidence of disruption of tumor vascularity with decreased microvessel density, depletion of endothelial cells and pericytes, and increased tumor cell apoptosis. These findings highlight the potential importance of AM and its receptors in the progression of CRC and support the conclusion that αAM treatment inhibits tumor growth by suppression of angiogenesis and tumor growth, suggesting that AM may be a useful therapeutic target.

## Introduction

Colorectal cancer (CRC) remains a leading cause of cancer-related death worldwide despite recent advances in adjuvant chemotherapeutic regimens. CRC progresses through a series of clinical and histopathological stages ranging from single crypt lesions through small benign tumors (adenomatous polyps) to malignant cancers (carcinomas) 1. The model of colorectal tumorigenesis includes several genetic changes that are required for cancer initiation and progression 2. The earliest and most prevalent genetic event yet identified in colorectal tumorigenesis is the disruption of a functional adenomatous polyposis coli (APC) complex due to a mutation of the APC gene or the β-catenin gene, leading to inappropriate activation of the Wnt signaling pathway 3,4. These results in nuclear accumulation of β-catenin, which associates with the T-cell factor-4, leading to transcription of genes involved in dedifferentiation, cell proliferation, and survival events involved in carcinogenesis.

Adrenomedullin (AM) is a multifunctional peptide with properties ranging from inducing vasorelaxation to acting as a regulator of cellular growth and angiogenesis 5–7. AM binds to and mediates its activity through the G-protein-coupled receptor calcitonin receptor-like receptor (CLR), with specificity for AM being conferred by the receptor activity-modifying protein-2 (RAMP2) and -3 (RAMP3) 8. The ability of CLR/RAMP2 and CLR/RAMP3 to respond with high affinity to AM implies the existence of two molecularly distinct AM receptors, respectively, referred as AM_1_ and AM_2_ receptors 9. Two other AM receptors (L_1_ and RDC1) with different affinities have already been described 6. AM is widely expressed in a variety of tumor types 10 and was shown to be mitogenic for human cancer cell lines including lung, breast, colon, glioblastoma, kidney, and prostate lineages in vitro 11–14. Several in vivo studies have shown a reduction of tumor angiogenesis and growth upon the treatment with neutralizing AM antibodies 11, AM receptor antagonist 15,16, or AM receptor RNA interference 17.

In the gastrointestinal tract, it has been reported that the expression of AM in the small intestine was localized in the mucosa and submucosa, but not in the muscularis or serosa 18. A very weak expression in the rodent colon at a distal site of the small intestine has been reported 18. In a normal colon, AM is able to regulate blood supply and protect the gut mucosa. In addition, it has been demonstrated that AM expressed in epithelial neuroendocrine cells and epithelial microvilli could exert effects such as antibacterial activity or may influence the absorption of nutrients 19,20. Immunoreactive AM has been reported in the human stomach, small intestine, and colon 21.

Although the expression of AM was reported in colorectal carcinoma cell lines Snuc 1 and DLD-1 22,23, little is known about AM and its receptors as well as its role in CRC. The frequency and distribution of AM and AM receptors expressions in tumors have not been previously reported and the role of AM in CRC is not completely understood. In this study, we investigated the expression of AM and its receptors in a large cohort of human CRC (primary tumors, lymph node, and distant metastasis) and used colorectal carcinoma cell line HT-29 to investigate the role of AM in cultured cells in vitro and in HT-29 xenografts in vivo.

## Materials and Methods

### Patient data and colon tumor samples

Two series of patients were enrolled in this study. They were consecutively treated for CRC in CHU Nord between 1992 and 2000. The eligibility criterion was a proven metastatic colorectal adenocarcinoma by histological biopsy. All patients signed an informed consent to participate and were over 18 years old. Surgical samples taken from CRC tumors or nonneoplastic tissue were obtained from the AP-HM Tumor Tissue Bank (ISO 9001:2008) at the CHU in Marseilles. Tumors were classified according to the International Union against Cancer (UICC) into different classical clinical stages 24. In the first series, frozen samples of colorectal tissues (*n* = 91) conserved in the AP-HM tumor bank from 45 women and 46 men were classified according to their clinical stages as follows: normal tissue (*n* = 30), stage I (*n* = 8), stage II (*n* = 32), stage III (*n* = 12), and stage IV (*n* = 9) and used to quantitate the AM mRNA levels.

The second series included CRC samples (*n* = 147) embedded in paraffin with clinical stage I (*n* = 21), stage II (*n* = 41), stage III (*n* = 44), and stage IV (*n* = 41) from 68 women and 79 women between 33 and 88 years old (mean = 65.7 years; SD = 13 years). These samples were used for tissue microarray (TMA) analysis and immunohistochemistry. Primary tumors and lymph node samples from 47 patients were also recovered in the second series.

### Cell culture

Human CRC cell line HT-29 was obtained from American Type Culture Collection (Rockville, MD) and maintained in minimum essential medium containing penicillin (50 U/mL), streptomycin (50 μg/mL), and glutamine (1 mg/mL), and supplemented with 10% fetal bovine serum. Cells were cultured under a moist 5%-CO_2_/95%-air atmosphere, and fed with fresh medium every 2 days, being routinely monitored for mycoplasma contamination (Roche Diagnostics, Meylan, France). Cells growing exponentially were harvested and prepared for RNA analysis and protein extracts. All culture media components were purchased from Invitrogen Life Technologies (Paris, France).

### RNA preparation and real-time quantitative RT-PCR

Total RNA was prepared from frozen CRC tumors, HT-29 cells, and HT-29 tumor xenografts, reverse transcribed to cDNA, and quantified as described 25.

### Development and characterization of polyclonal anti-human AM antibody

The polyclonal antibody against human AM was developed by use of the synthetic peptide corresponding to the entire AM_1–52_ amide peptide (Bachem, Weil am Rhein, Germany) as described 11. Female New Zealand rabbits received injections at multiple subcutaneous sites with 300 μg of synthetic peptide emulsified with complete Freund's adjuvant. The rabbits were subsequently further immunized at 2.5 week intervals with 120 μg of AM_1–52_ amide emulsified with incomplete Freund's adjuvant. The antisera obtained after the fourth booster injection were screened for anti-AM activity, and then affinity purified on rProtein A Sepharose Fast Flow columns (GE Healthcare, Vélizy-Villacoublay, France). The anti-AM polyclonal antibody (purified IgG) showed very low cross-reactivity (<7%) with AM-related peptides such as AM_22–52_ amide, AM_26–52_ amide, and AM_13–37_. Calcitonin, CGRP_1–37_ amide, CGRP_8–37_ amide, and amylin showed insignificant anti-AM antibody binding (<0.1%) despite some homology with AM. We also demonstrated that anti-AM antibody blocked the binding of ^125^I-AM to its cell-surface receptor on HT-29 cells in a dose-related manner.

### Immunohistochemistry of AM, CLR, RAMP2, and RAMP3 proteins

Tumor specimens were frozen on dry ice/butane, and stored at −80°C. Frozen sections (6 μm) were cut on a Leica cryostat. Sections of each specimen were stained using hematoxylin and eosin (H&E). Immunohistochemistry was carried out using the Vectastain Elite ABC Kit (Vector Laboratories, Burlingame, CA). Optimal dilution for rabbit anti-AM polyclonal antibody (referred here as αAM), anti-CLR (αCLR), anti-RAMP2 (αRAMP2), and anti-RAMP3 (αRAMP3) developed and characterized following the same protocol described for the generation of anti-AM antibody 5,15 were respectively used at dilution of 1:1000, 1:3000, 1:2000, and 1:1500. Detection was carried out using DAB chromogen. As a control for immunostaining, the antibodies preabsorbed by human synthetic AM peptide (50 μmol/L; Bachem), CLR, RAMP2, and RAMP3 peptides (50 μmol/L synthesized in the laboratory) were used instead of the primary antibodies.

### Tissue microarray construction, immunohistochemistry, and image analysis

Tissue microarray construction and analysis were performed as previously described 26. Sections of paraffin-embedded samples of human CRC specimens were analyzed using the automate image analyzer as described 27.

### Cell proliferation and invasion assays

The effects of AM, AM_22–52_, αAM (purified IgG), αCLR, αRAMP2, and αRAMP3 on cell proliferation were examined at the indicated time points as described 11. The invasion was assessed using a modified Boyden chamber assay as previously described 5.

### Peptide extraction and AM radioimmunoassay

Extraction of proteins and immunoreactive-AM (ir-AM) radioimmunoassay (RIA) were performed as previously described 12.

### Experimental protocol for animals

Animal work was carried out in the animal facility of the School of Medicine according to the institutional animal welfare guidelines. Athymic NMRI (nu/nu) nude mice (Harlan, Gannat, France) were maintained in a sterile environment with a daily 12 h light/12 h dark cycle. HT-29 cells (3 × 10^6^) were s.c. injected in the right flanks of nude mice. Tumors were measured with a dial-caliper, and volumes were determined using the formula width × length × height × 0.5236 (for ellipsoid form). After 20 days, when the primary tumors were 300–500 mm^3^ in size, animals were randomly divided into two groups. One group (*n* = 20) received intraperitoneal injection of the αAM (350 μg of purified IgG) every 3 days. The amount of αAM was determined based on the data of preliminary experiments in which increasing amounts of αAM (100, 200, 350, 500, 800 μg) were used to determine the best concentration of αAM inhibiting xenograft growth in vivo. As control, one group (*n* = 10) received a rabbit control-IgG (350 μg) of irrelevant specificity. Mice were sacrificed at the indicated time.

### Immunohistochemical analysis

All tumor xenografts were excised, fixed in 10% (v/v) formalin, and processed for immunohistochemical analysis. Paraffin blocks were cut to 6 μm sections and stained with H&E for morphology evaluation. Immunohistochemistry was carried out using the Vectastain Elite ABC Kit (Vector Laboratories). Sections were incubated with anti-von Willebrand factor (anti-vWF) (1:400; Dako, Trappes cedex, France), or anti-α-Smooth Muscle Action (anti-α-SMA) (1:80; Dako), and subsequently with fluorochrome (Alexa 488 or Alexa 647)-conjugated secondary antibodies (Invitrogen Life Technologies). To assess a programmed cell death, tissue sections were evaluated using Mab F7-26 to detect single-strand DNA (AbCys, Paris, France). For nonimmunofluorescence staining, detection was carried out using a DAB chromogen, which resulted in a positive brown staining. Sections were counterstained with hematoxylin. As a control for immunohistochemistry, normal rabbit or mouse serum was used instead of the primary antibodies.

### Statistical analysis

Data are expressed as mean ± SEM from at least three independent experiments. One-way analysis of variance (ANOVA) or Fisher's protected least significant difference test (Statview 512; Brain Power Inc., Calabasas, CA) was used for statistical analysis. *P* < 0.05 was considered significant and is indicated with asterisk in the figures. A double and triple asterisk, respectively, indicates *P* < 0.01 and *P* < 0.001.

## Results

### Expression of AM mRNA in human CRC

Total RNA from human colorectal normal tissue and human CRC was prepared to assess steady-state levels of AM mRNA transcript. Real-time quantitative RT-PCR analysis was performed on colorectal stage 0 fragments (*n* = 30) and tumor fragments of the 61 CRC that present samples with clinical stage I (*n* = 8), stage II (*n* = 32), stage III (*n* = 12), and stage IV (*n* = 9). Quantification of AM mRNA transcripts revealed high levels of AM mRNA in CRC clinical stages II, III, and IV, compared with colon stage 0 tissue and CRC clinical stage I (Fig. 1). The mean level of AM mRNA expression was 364 ± 46 fg/pg GAPDH mRNA in colorectal normal tissue (mean ± SEM), whereas it was, respectively, 457 ± 133, 810 ± 156, 825 ± 151, and 1072 ± 265 fg/pg GAPDH mRNA for CRC stages I, II, III, and IV (Fig. 1). AM mRNA levels determined in CRC stages II, III, and IV were significantly higher when compared with colorectal stage 0 tissue (*P* < 0.0078, *P* < 0.0009, *P* < 0.0005, respectively). Omission of the reverse transcriptase eliminated the signal, indicating that it was not linked to contaminating genomic DNA (not shown).

**Figure 1:** AM mRNA levels in normal and tumor colorectal tissues. Total RNA, DNA free, prepared from normal colon tissue and colorectal cancer (CRC) at different clinical stages (I–IV) were transcribed to cDNA and subjected to real-time quantitative RT-PCR for the estimation of relative AM mRNA to GAPDH mRNA ratios. Each bar represents the mean ± SEM of two independent assays in triplicate. The asterisk indicates that the values for CRC (clinical stages, II, III, and IV) are significantly different from the values of normal tissue and stage I of CRC (*P < 0.05; **P < 0.01; ***P < 0.001).

### Immunohistochemistry of AM, CLR, RAMP2, and RAMP3 proteins

Adrenomedullin, CLR, RAMP2, and RAMP3 proteins immunodetections are shown in Figure 2. AM labeling was slightly detectable in the majority of the epithelial compartment of the crypts (Fig. 2a). Positive stained cells are observed in the stroma that could be macrophages, mast cells, and leukocytes (Fig. 2a). Well-differentiated cancer specimens displayed overt and strong AM labeling of epithelial cells, but not stromal cells (Fig. 2b). A higher degree of labeling was observed in poorly differentiated specimen with a clear increase in distant metastasis tissue (Fig. 2c and d). CLR, RAMP2, and RAMP3 immunostaining was barely detectable in the colonic epithelia of the crypts in normal tissue (Fig. 2e, i, and m). Cancer specimens displayed a strong staining for CLR, RAMP2, and RAMP3 of the epithelial compartment of the crypts in the well-differentiated adenocarcinomas (Fig. 2f, j, and n). The same labeling is observed in poorly differentiated (Fig. 2g, k, and o) and distant metastasis tissues (Fig. 2h, l, and p). Positive AM staining was completely abolished by preabsorption of the antibody with 50 μmol/L synthetic AM (Fig. 2q, r, s, and t) or CLR, RAMP2, RAMP3 peptides (not shown).

**Figure 2:** Immunohistochemistry for AM, CLR, RAMP2, and RAMP3 of the normal and tumor colorectal tissues. In normal tissue, AM immunoreactivity is observed in the cytoplasm of the epithelial cells and some cell types in the stroma (a). Positive immunoreactivity against CLR (e), RAMP2 (i), and RAMP3 (m) in epithelial cells is very weak in normal tissue. In well-differentiated colorectal cancer specimens, a far more intense labeling of epithelial cells is observed. In poorly differentiated and distant metastasis, a heavily labeled adenocarcinomatous structure can be observed. AM immunoreactivity is completely canceled by the antibody preabsorbed with 50 μmol/L AM peptide (q, r, s, and t). Magnification: ×10. AM, adrenomedullin; CLR, calcitonin receptor-like receptor; RAMP2, receptor activity-modifying protein-2; RAMP3, receptor activity-modifying protein-3.

Adrenomedullin immunoreactivity was revealed in the apical side cytoplasms of surface columnar epithelia of the human colonic mucosa and in the musculus (Fig. 3a). Interestingly, in the normal colon, AM immunoreactivity was also detected in neuroendocrine cells (Fig. 3b) as previously reported 14.

**Figure 3:** Adrenomedullin (AM) immunoreactivity of the human colonic mucosa. Immunoreactivity for AM is observed in the apical side cytoplasm of the surface epithelia and at the luminal surface (a). Positive immunoreactivity for AM is also noted in neuroendocrine cells (b). Magnification ×20.

### TMA of AM, CLR, RAMP2, and RAMP3 proteins

To further investigate the prognostic value of AM, CLR, RAMP2, and RAMP3 expression, we used automatized quantitative image analysis on TMA. The data demonstrate that AM is expressed in all colorectal primary tumors and the staining quantification showed no significant changes between patients with different grades (Fig. 4a), either in the absence of negative (N0) or in the presence of positive (N+) lymph node (Fig. 4b); nor between clinical stages (I–IV) (Fig. 4c). Interestingly, an increase in AM staining was found in lymph node and distant metastasis when compared with primary tumors (Fig. 4d). Similarly, a significant increase in the staining was obtained for CLR, RAMP2, and RAMP3 proteins (*P* < 0.001; Fig. 4e). There was no difference between lymph node and distant metastasis. On the contrary, TMA analysis of primary tumor tissue and associated lymph node (N+) for each individual patient (*n* = 47) showed a highly significant increase of AM as well as CLR, RAMP2, and RAMP3 staining in lymph node when compared with primary tumor tissue (*P* < 0.001; Fig. 4f and g).

**Figure 4:** Statistical analysis of αAM and αAMR staining on TMA slices. ANOVA analysis of TMA-1 staining of cohort of patients (*n* = 147) according to histological grade T1, T2, T3, T4 (a); node status associated (N+) or not (N0) with metastatic process (b); and the clinical stages (I, II, III, IV) (c). TMA analyses for the expression of AM and AMR (CLR, RAMP2, and RAMP3) were quantified in tumor (T), node (N), and metastasis (M) (d, e). Expression of AM (f) and AMR (g) obtained with TMA analysis with tumors and nodes samples issued from the same patients (*n* = 47). Data demonstrate a clear increase of AM, CLR, RAMP2, and RAMP3 expression in nodes versus tumors (***P < 0.001). TMA, tissue microarray; AM, adrenomedullin, αAM, anti-AM; αAMR, anti-AM receptors, CLR, calcitonin receptor-like receptor; RAMP2, receptor activity-modifying protein-2; RAMP3, receptor activity-modifying protein-3.

### Expression of AM and regulation by hypoxia in HT-29 cells

The expression of AM and its receptors in colorectal carcinomas suggest that the AM system might play a role in promoting tumor growth in situ. Accordingly, we used HT-29 cells to have more insight in the role of AM system in CRC. Quantitative RT-PCR analysis demonstrated that HT-29 cells express AM mRNA (Fig. 5a) and interestingly, sixfold increase of AM mRNA expression was observed under hypoxia (Fig. 5a). RIA demonstrated a clear increase of secreted immunoreactive-AM (ir-AM) by HT-29 cells under hypoxia versus normoxia (48 ± 2 pg/mL/h vs. 26 ± 7 pg/mL/h). Accordingly, the intracellular ir-AM showed an increase under hypoxia versus normoxia (12.32 ± 0.61 pg/μg protein/h vs. 7.41 ± 1.28 pg/μg protein/h).

**Figure 5:** AM stimulates proliferation and invasion of HT-29 cells in vitro. (a) Expression of AM mRNA in HT-29 cells. Total RNA (1 μg) DNA-free prepared from HT-29 cells was reverse transcribed into cDNA and subjected to quantitative RT-PCR for the estimation of relative AM to GAPDH mRNA ratios. Error bars indicate the SEM. The asterisks indicate that the value in HT-29 cells under hypoxia is significantly different from the HT-29 cells under normoxia in vitro (***P < 0.001). (b) For proliferation assays, tumor cells were seeded at the density of 2 × 10^3^ per well in 12 multiwell plates in the presence of ITS medium. AM at 10^−7^ mol/L, αAM (30 μg/mL), combined αCLR/αRAMP2 or αCLR/αRAMP3 (30 μg/mL), AM_22–52_ at 10^−6^ mol/L, and control-IgG (30 μg/mL) were added for 6 days treatment. For each treatment, six wells were prepared for MTT assays. Bars represent SEM of three independent experiments. **P < 0.01; ***P < 0.001. (c) for invasion, HT-29 cells (3 × 10^4^) were seeded on a Matrigel layer in a Boyden chamber assay. HT-29 cells were preincubated for 30 min with 15 μg/mL each of αCLR/αRAMP2 or αCLR/αRAMP3, AM_22–52_ at 10^−6^ mol/L or control-IgG. AM at indicated concentrations was added in the lower wells. Cells migrating through the filter were counted after 24 h. Data are expressed as the percentage of migrated cells in 10 high-power fields and are the means of three independent experiments each performed in triplicate. Bars represent SEM. ***P < 0.001 compared to control. AM, adrenomedullin; αAM, anti-AM; αCLR, anti-calcitonin receptor-like receptor; αRAMP2, anti-receptor activity-modifying protein-2; αRAMP3, anti-receptor activity-modifying protein-3.

### AM stimulates HT-29 cells growth and invasion in vitro

The expression of AM and its receptors in CRC tissues as well as in cell lines suggests that AM might be involved in CRC cell growth by an autocrine/paracrine mechanism. AM at 10^−7^ mol/L stimulated the proliferation of HT-29 cells by 20% (*P* < 0.01) after 6 days of treatment (Fig. 5b). To test the autocrine hypothesis, HT-29 cells were treated with 30 μg/mL of αAM, αCLR/αRAMP2, or αCLR/αRAMP3 (purified IgG) to determine their effect on the in vitro growth of the HT-29 cells. The inhibition of proliferation reached up to 70% (*P* < 0.001) and 80% (*P* < 0.001) by 6 days of treatment, respectively, when compared to control (Fig. 5b). In contrast, control IgG (30 μg/mL) of irrelevant specificity (Fig. 5b) showed no inhibition of proliferation. To confirm that endogenous hAM produced by the HT-29 cells acts as an autocrine growth factor, HT-29 cells were incubated for up to 6 days with the AM antagonist AM_22–52_ at 10^−6^ mol/L. In the presence of AM_22–52_, inhibition of cell growth reached up to 70% (*P* < 0.001) when compared with control cells (Fig. 5b). Taken together, these observations support that AM acts as an autocrine growth factor via AM_1_ and AM_2_ receptors to stimulate HT-29 cells proliferation.

To further investigate the influence of AM on CRC cell function, the invasive capacity of HT-29 cells in response to AM was investigated by measuring the invasion of a Matrigel layer in a Boyden chamber assay. AM induced a dose-dependent increase in HT-29 cells invasion through Matrigel coating of the membrane (*P* < 0.005) (Fig. 5c), with a threefold increase in the number of migrated cells was obtained with AM at 10^−14^ mol/L (Fig. 5c). Preincubation of HT-29 cells with αCLR/αRAMP2, αCLR/αRAMP3, or AM_22–52_, completely blocked the invasion induced by AM indicating that the AM_1_ and AM_2_ receptors are involved in the response to AM (Fig. 5c). Preincubation of the cells with control IgG did not block the induced effect of AM on invasion (Fig. 5c). These observations demonstrate that AM induces HT-29 cells invasion via the AM_1_ and AM_2_ receptors.

### αAM inhibits growth of HT-29 tumor xenograft

To assess the potential therapeutic value of αAM, athymic nude mice bearing established HT-29 tumor xenografts (>300 mm^3^) were treated with αAM or a rabbit control IgG of irrelevant specificity. Treatment was administered by i.p. injection every 3 days and tumor growth was monitored as a function of tumor volume through the time of therapy. The growth of HT-29 xenografts was significantly inhibited by the αAM when compared with control group (Fig. 6a). After a 40 day treatment period, a group of animals (*n* = 8) were sacrificed, and tumor size and vascularity were assessed. Tumors from αAM-treated animals appeared pale with diminished vasculature, whereas large tumors with extensive vascularization were observed in control groups. The mean tumor weights in the control and in the αAM-treated groups were 2.8 g versus 0.8 g at 60 days of treatment.

**Figure 6:** Treatment with anti-adrenomedullin (αAM) inhibits growth of HT-29 xenograft in vivo. HT-29 tumor xenografts were established by injecting 3 × 10^6^ HT-29 cells subcutaneously into the right flank of athymic (nu/nu) nude mice. (a) Tumors were allowed to reach 300–500 mm^3^ in size, mice received i.p. injections of αAM (350 μg/mouse) every 3 days. Control mice were treated with 350 μg/mouse of nonimmune control-IgG. Tumor size was measured every 3 days. In animals treated with αAM, the size of tumors was significantly smaller. (b and d) Microphotographs of immunofluorescence and immunohistochemical-stained tumor sections for von Willebrand factor (vWF) (red), α-SMA (green), and single-strand DNA(ssDNA) in control and αAM-treated tumors. DAPI-stained nuclei are blue. Scale bars = 30 μm. (c) Quantitative assessment of the cells density that stained positive for vWF and α-SMA through a microscope. NIH image 1.62 software was used for analysis. Values are means ± SD; *n* = 8. ***P < 0.001. (e) Cells undergoing apoptosis were determined using Mab F7-26, which stained ssDNA. Values are means ± SD; *n* = 6, ***P < 0.001.

Histological examination of αAM-treated tumors for 60 days showed a significant decreased vessel density when compared with control IgG-treated group (Fig. 6b). Immunostaining of tumors with antibodies for vWF demonstrated that αAM-treated tumors were noticeably less vascular than control tumors (Fig. 6b). Costaining with anti-vWF and anti-α-SMA antibodies demonstrated that both cell types are sparse, and the vascularization is deeply disrupted and characterized by an overall reduction of endothelial cells and pericytes (Fig. 6b). In contrast, control IgG-treated tumors showed a well-organized vascularization (Fig. 6b). Quantification of vWF-stained endothelial cells demonstrates a clear decrease of vWF-positive cells in αAM-treated tumors when compared with control IgG-treated tumors (*P* < 0.001; Fig. 6c). Interestingly and despite the fact that the apoptosis labeling is heterogeneous among the tumors, the apoptotic index of the αAM-treated tumors was two- to threefold higher than the control tumors (*P* < 0.01; Fig. 6d and e).

## Discussion

In this study, we investigated the expression of AM in normal and CRC tissues and its potential role as an autocrine/paracrine growth factor to promote CRC growth in vitro and in vivo. In the normal colon tissue, our immunohistochemical study demonstrates that AM is located in the cytoplasm of epithelia of the crypts and in the colonic surface epithelia in addition to neuroendocrine cells. The surface epithelium serves as a protective barrier between the host and the luminal environment. An immunopositive reaction to AM was observed at the luminal surface, which could indicate that AM was actually released from the colonic epithelia into the lumen. These lines of evidence suggest that AM may play some functional roles such as contribution to the mucosal defense system without ruling out some unrecognized roles in the digestive system. Many authors have reported that AM has bactericidal activity against Gram-positive and -negative bacterial strains 19,20.

The expression of AM and its receptors in CRC tissue strongly suggest that AM might be involved in CRC progression. Real-time quantitative RT-PCR demonstrated a significant increase in the expression of AM mRNA levels in late clinical stages compared with stage I of CRC. Immunohistochemical analysis localized a high staining of AM and AM receptors in the carcinomatous epithelial compartment of colorectal tumors when compared to a detectable staining in epithelial cell from normal tissue localized in the crypts. The expression of AM, CLR, RAMP2, and RAMP3 in a large number of samples of human CRC was assessed by TMA analysis. The data demonstrated the presence of AM and its receptors in the vast majority of colorectal adenocarcinomas of different clinical stages. The amount of AM staining in colorectal tumor tissues represents a balance among synthesis, storage, degradation, and secretion. The dissociation between levels of AM mRNA and AM staining in late clinical stages may reflect an increase of secretion rate of ir-AM and/or altered translational efficiency for AM mRNA. Interestingly, a higher expression of AM and its receptors was found in the CRC-associated node (*n* = 47) when compared with a primary colorectal tumors, strongly suggesting that AM might be involved in the colorectal metastasis.

The degree of AM expression has been associated with lymph node metastasis in breast cancer 28,29. In pancreatic adenocarcinoma, the median AM mRNA expression levels were higher in lymph node-positive compared with lymph node-negative patients 30. Lymph node metastasis is a sensitive indicator of poor prognosis in patients with CRC 31,32,33, but even in node-negative patients, approximately 10–20% patients suffer from relapse in <5 years 34. Recently, Uemura et al. 35 reported that AM was a novel independent prognostic factor for CRC with no correlations between AM expression and lymph node metastasis.

Previous studies have demonstrated the ability of reduced oxygen tension to mediate elevations in AM message/protein expression in several animal and cell systems 23. Nakayama et al. 23 have demonstrated that hypoxia stimulates AM expression in human colorectal carcinoma cell line, DLD-1. This study demonstrates that hypoxic conditions induced an increase of AM expression in HT-29 cells. These data suggest that the resulting reduction in tissue oxygen tension may lead to an increased expression of AM mRNA in colorectal tumors. Interestingly, a recent study reported that the expression of AM correlated with hypoxia-inducible factor-1α in vivo samples from a cohort of 373 CRC patients 35.

The presence of AM and AM receptors (AM_1_ and AM_2_) opens up the possibility for AM to be an autocrine/paracrine growth factor in CRC. This hypothesis is supported by the data showing that exogenous AM stimulates HT-29 cell growth. Proliferation assays revealed that a neutralizing αAM and αAMR could significantly suppress cell growth of HT-29 cells. The inhibition by αAM could be reversed by the addition of the exogenous AM, thus, the inhibition of cell growth by αAM and αAMR in vitro was most likely the result of blocking the autocrine/paracrine effects of immunoreactive AM synthesized and secreted by the colorectal carcinoma cells. These observations indicate that colorectal carcinoma cells are able to respond to AM in ways that would be expected to further promote cell and tumor growth. Our conclusion that AM can act as an autocrine/paracrine growth factor in colorectal carcinomas is in agreement with the previously reported data in other forms of cancer where AM may act in the same manner 11,12–17,30.

To extend the in vitro observations, in vivo experiments were performed. Our results demonstrated that the αAM significantly suppresses the growth of established HT-29 tumor xenografts. After 2 months of treatment, tumors in mice treated with control-IgG grew progressively to a size that led to sacrifice, whereas the volume of the αAM-treated tumors decreased by 95% after 80 days of treatment. The immunohistological analysis of tumors from αAM-treated animals showed a clear decrease in microvessel density with 80% reduction of endothelial cells and pericytes within the tumor, confirming the role of AM in endothelial cells and pericytes activation and/or recruitment. These data demonstrate that AM is involved in neovascularization and/or vessel stabilization. AM signaling is of particular significance in endothelial cell biology because the peptide protects these cells from apoptosis 36,37, promotes angiogenesis and vascular stabilization 5,38, and affects vascular tone and permeability 39. Our findings are consistent with the previously reported data involving AM in tumor angiogenesis through CLR/RAMP2 and CLR/RAMP3 5,15,38. Previously, our group reported that targeting AM receptors with systemic delivery of neutralizing antibodies inhibits tumor angiogenesis and suppresses growth of colorectal carcinoma HT-29, U87 (glioblastoma), and A549 (lung cancer) tumor xenografts in mice 15.

In summary, our study demonstrates the relevance of AM and its receptors CLR/RAMP2 and CLR/RAMP3 in CRC. Our data strongly suggest that AM is involved in the progression of colon cancer. Targeting AM system by αAM treatment inhibits tumor growth by suppression of angiogenesis and tumor growth, suggesting strongly that AM may be a useful therapeutic target.
